The article "Analysis of Urban Residents' Consumption Behavior and Influencing Factors of Ecological Agricultural Products in the Post-Pandemic Era of COVID-19" was retracted in 2022. Reason: concerns about the peer review.

# Analysis of Urban Residents' Consumption Behavior and Influencing Factors of Ecological Agricultural Products in the Post-Pandemic Era of COVID-19

**DOI:** 10.1155/2022/8382247

**Published:** 2022-05-14

**Authors:** Ximing Chen, Jie Shang

**Affiliations:** School of Economics and Management, Northeast Forestry University, Harbin, 150040 Heilongjiang Province, China

## Abstract

Based on consumer survey data in the post-pandemic era of COVID-19, a binary Logit model was used to analyze the consumers' consumption behavior and the influencing factors of ecological agricultural products in the post-pandemic era. The results showed that: family size, average annual household income, gender, and education level would not affect the consumers' behavior in purchasing ecological agricultural products after the pandemic; age and whether consumers have purchased agricultural products before had a significant negative impact on consumption behavior; the degree of consumers' skepticism about agricultural products in the market after the pandemic had a significant positive impact on their purchase behavior. According to the analysis results, it is proposed that: we should vigorously develop the connection between agricultural socialized service industry and large supermarkets, improve the online and offline sales model of ecological agricultural products, establish an ecological agricultural product service platform, and enhance the scientific and technological researches and their application to ecological agricultural products.

## 1. Introduction

The novel coronavirus pneumonia pandemic in 2020 brought a hitherto unknown public health crisis, and the agricultural food systems in various countries are facing major challenges. In the context of the novel coronavirus pneumonia, the prices of agricultural products have been rising consistently. From the second half of 2020 to March 2021, the international food price index had risen by more than 27.3%. In the face of rising prices, people have turned their attention to certified, pollution-free ecological agricultural products. Therefore, it is significant to explore the behaviors and influencing factors of residents' consumption of ecological agricultural products in the reconstruction of the agro-food system in the post-pandemic era.

People's cognition level, consumption willingness and purchase behavior of ecological agricultural products are all affected and restricted by many factors. After the pandemic, what are the residents' awareness level, consumption willingness and purchasing behavior of ecological agricultural products like in the post-pandemic era? Are consumers' purchasing decisions consistent with their awareness and purchase intentions? What are the factors affecting residents' purchasing behavior of ecological agricultural products? Solving these problems will be of great significance to the production and development of ecological agricultural products after the pandemic. This paper conducted a questionnaire survey with a discrete random sampling method, analyzed residents' consumption behaviors and influencing factors of ecological agricultural products in the post-pandemic era through a binary Logit model, dentified the key factors that influence the consumption decision of ecological agricultural products and explained the inconsistency between consumer wishes and purchasing behavior.

The article "Analysis of Urban Residents' Consumption Behavior and Influencing Factors of Ecological Agricultural Products in the Post-Pandemic Era of COVID-19" was retracted in 2022. Reason: concerns about the peer review.

## 2. Relevant Literature and Research Hypotheses

### 2.1. Ecological Agricultural Product Concept

Agricultural products generally refer to the unprocessed or primary processed food, vegetables, milk, eggs, fungi, aquatic products, etc. Ecological Agriculturel products are emerging concepts derived from the continuous development of traditional agricultural products. Based on agricultural products, they involve multi-disciplinary fields such as agricultural economics, ecological agriculture, and environmental science. In a narrow sense, ecological agriculture products include ecological agricultural products that use agricultural green production materials as raw materials and undergo a series of processing procedures on the raw materials. Compared with traditional agricultural products, ecological agricultural products have higher nutritional value and commercial value, and belong to high-end products in agricultural products.

### 2.2. Research on Ecological Agricultural Products

At present, countries have not reached a consensus on the concept of ecological agricultural products. In the United States, the United Kingdom and other countries, it's generally called organic agricultural products; in Japan, it's called natural agricultural products; in Sweden and Finland, it's called ecological agricultural products [1]. The Food and Agriculture Organization of the United Nations has elaborated on organic agriculture and it believes that sustainable environmental development and the most ecological benefits can be achieved through green production and material recycling, consumption restriction of energy and materials, as well as pest prevention and controlling. The optimized ecological production system is “organic agriculture”. Farm products produced according to its standards are called “organic agricultural products” [2]. China has also defined the concept of ecological agricultural products, which generally refers to the adherence to strict protection and improvement of the agricultural production environment. According to the objective laws of ecology and ecological economics, combined with modern green agriculture and ecological agricultural production technology, and under the intensive management mode, the nutritious, harmless and healthy ecological agricultural products that meet the national ecological agricultural product quality standards can be produced [3].

The article "Analysis of Urban Residents' Consumption Behavior and Influencing Factors of Ecological Agricultural Products in the Post-Pandemic Era of COVID-19" was retracted in 2022. Reason: concerns about the peer review.

### 2.3. Research on Consumer Purchasing Behavior

The research on consumer behavior began in the 1960s. Consumer behavior is affected by consumers' purchase intentions. As a kind of willingness, the willingness to consume also belongs to a category studied by psychology and it generally refers to the subjective thinking of an individual about food. Feng Jianying systematically summarized the influencing factors of consumers' purchase intentions and believed that consumers' own attributes (including gender, age, occupation, income and education level), internal characteristics of products (including product value standards, use value and quality), and external factors of products (including store environment, design style and shopping experience) will have an impact on consumers' purchase intentions [4]. Researches on the attributes of consumers believe that gender, age, and education level play a significant role in the consumption of ecological agricultural products. Taking Tianjin as an example, Zhang Xiaoyong and others found that the income of residents has little effect on the purchase of ecological agricultural products, while gender, age and education level have significant effects on it [5]. Aiming at exploring the internal characteristics of products, Yuan Fengbai (2017) believed that sales promotion activities and gift promotion activities have a positive effect on consumers' purchase of green agricultural products [6]. In the research on the external factors of products, Zhang xuemu and Wang Xining (2019) in the article “the impact of ecological labels on the purchase intention of green products - taking consumers' perceived value as the intermediary” believed that the ecological labels play a complete intermediary role in consumers' purchase intention of green production, and environmental value plays a partial intermediary role in it [7].

### 2.4. Research on the Purchase Intention of Ecological Agricultural Products

Due to the differences in the concept of ecological agricultural products, foreign researches on the purchase intention and behavior of ecological agricultural products mainly focus on organic agricultural products. Elif and Bulent believed that safety, environmental protection, and product quality are important factors that affect consumers' choices of organic agricultural products [8]. Michaelidou N, Hassan LM analyzed consumers' attitudes and willingness to organic agricultural products through mechanism models. The results showed that consumer moral identity will affect consumption willingness, and the core element of its influence is consumers' attention to organic agricultural products [9]. Domestic researches on ecological agriculture started relatively late. Through the construction of comprehensive evaluation indicators for trust, Yang Xiaoli and others studied the factors affecting consumer trust in organic agricultural products, including system, ecological environment, corporate credibility, and corporate social influence [10]. Xie Tianyun and others analyzed the consumption behavior of residents in Zhangjiakou City. They believed that consumers have no trust in ecological agricultural products at this stage, and the price factors of ecological agricultural products seriously hinder consumers from purchasing behavior. At the same time, it is still affected by internal attributes including age, education level, family demographic structure, household monthly income and other personal attributes, as well as external conditions such as trust in products, ease of purchase, and consumer satisfaction [11]. On the whole, the existing researches mainly focus on surveys of a certain city, studying consumers' awareness of ecological agricultural products, purchase intention and influencing factors. Due to the impact of the novel coronavirus, this article used a questionnaire survey based on existing researches to analyze the residents' consumption behavior of ecological agricultural products and the influencing factors under the special circumstances of the post-pandemic era.

The article "Analysis of Urban Residents' Consumption Behavior and Influencing Factors of Ecological Agricultural Products in the Post-Pandemic Era of COVID-19" was retracted in 2022. Reason: concerns about the peer review.

Based on the research of existing related literature, this article put forward the following hypotheses about consumers' consumption behavior of ecological agricultural products in the post-pandemic era:

**Hypothesis 1 .**

The more family members there are, the more ecological agricultural products are consumed.

**Hypothesis 2 .**

The higher the household income level is, the more ecological agricultural products are consumed.

**Hypothesis 3 .**

The higher the education level of consumers is, the more they understand about the novel crown pneumonia, the more ecological agricultural products are consumed.

**Hypothesis 4 .**

Since the consumption level of men is higher than that of women, men buy more ecological agricultural products than women.

**Hypothesis 5 .**

The elderly pay more attention to the quality of agricultural products, so they purchase more ecological agricultural products.

**Hypothesis 6 .**

People who have purchased ecological agricultural products before will increase their purchase of ecological agricultural products after the pandemic.

**Hypothesis 7 .**

People who are skeptical about food safety after the pandemic will pay more attention to the safety of ecological agricultural products, and they will increase their purchases of ecological agricultural products.

## 3. Data Source and Statistical Description

### 3.1. Data Source

This study adopted the method of questionnaire survey. In October 2021, the questionnaire was distributed on the Internet, and a total of 446 complete questionnaires were collected. The questionnaire consists of four parts: the first part is the characteristics of consumers, including gender, age, marital status, education level and occupation; the second part is the family characteristics of consumers, including family members and family income; the third part is the ecological perception of consumers, including whether they understand ecological agricultural products, the degree of concern for ecological agricultural products, and their skepticism towards agricultural products after the pandemic; the fourth part is the consumer behavior of ecological agricultural products, including the choice of locations to purchase ecological agricultural products, the consumption behavior of ecological agricultural products after the pandemic, and the decisive factors for purchasing agricultural products.

### 3.2. Statistical Description

#### 3.2.1. Consumer's Own Characteristics

As can be seen from Table 1, among the consumers surveyed, males account for 19.06% and females account for 80.94%; the ages of consumers are concentrated between 41 and 60, and they are mostly married; they mainly hold college degree or bachelor degree; most of them work in state-owned enterprises and public institutions.

#### 3.2.2. Family Characteristics of Respondents

It can be seen from Table 2 that mostly, there are 3 to 4 persons in the modern family, accounting for 76.46% of the sample population, and families with more than 5 persons account for 5.61%; the average annual incomes ranging from 30,000 to 50,000 yuan and 50,000 to 100,000 yuan account for 28.92% and 30.49%, respectively, and also a large proportion of less than 30,000 yuan account for 22.87%, who are mainly employees from rural areas, private enterprises and students, as seen in Table 1.

#### 3.2.3. Consumers' Ecological Perception

The perceptions of ecological agricultural products, consumption experience and satisfaction degree of the consumers surveyed are shown in Table 3. 93.95% of the surveyed consumers are aware of ecological agricultural products; majority of them express average concern about ecological agricultural products; only 14.57% are very concerned about them. Regarding the safety of agricultural products in the market after the novel coronavirus pneumonia, most people think they are safe, accounting for 46.84%, but 44.39% are skeptical about the safety of agricultural products in the market, which reveals that people are getting higher and higher standards of living. Among the surveyed consumers, 73.77% of them have purchased ecological agricultural products before, and they are basically satisfied afterward; only 2.47% of them consume more than three times a week, most of whom are middle-aged people between 30 and 59 who undertake the task of purchasing agricultural products.

The article "Analysis of Urban Residents' Consumption Behavior and Influencing Factors of Ecological Agricultural Products in the Post-Pandemic Era of COVID-19" was retracted in 2022. Reason: concerns about the peer review.

#### 3.2.4. Consumers' Ecological Agricultural Products Consumption Behavior

This research on consumer behavior of ecological agricultural products mainly investigated the consumption location, whether the consumption behavior would change due to the pandemic, and consumers' acceptable price fluctuations for ecological agricultural products (see Table 4). The results show that consumers surveyed are more accustomed to buying agricultural products in large supermarkets, with consuming online or buying products grown by private farmers as other options; after the pandemic, 73.54% of them are not willing to change the place where they bought agricultural products; and more than half of them will increase the purchase of ecological agricultural products after the pandemic, of which 76.68% are interested in the supply process of ecological agricultural products. On the premise of understanding ecological agricultural products, the number of consumers buying ecological agricultural products has increased by 8.52%, while only 1.79% of people can accept ecological agricultural products, whose prices are 31%-50% higher than the ordinary ones. It can be seen from the determinants of the purchase of ecological agricultural products that people are more concerned about the safety, price and nutrition of ecological agricultural products, and pay less attention to services, brands and packaging.

## 4. Measurement Analysis

### 4.1. Model Setting

Consumers have “choice” and “no choice” when they choose to purchase ecological agricultural products after the pandemic. Every consumer makes the best choice based on a rational comprehensive balance of various factors. Therefore, this is a typical dual decision-making problem. This article used the dual Logit regression model to analyze the factors affecting consumers' behavior in purchasing ecological agricultural products after the pandemic. The model is set as follows:

(1) $$\begin{array}{c} P=F\left(\left.y=1\right|X\right)=\frac{1}{1+e^{-y}} \end{array}$$

The y in formula (1) represents the consumer's choice to purchase ecological agricultural products after the pandemic. When a consumer chooses to purchase ecological agricultural products, y =1; otherwise, y =0. P represents the probability of consumer choice behavior; *x*_*i*_(*i* = 1, 2, ⋯⋯*n*) is a factor that may affect consumer choice behavior. In formula (1), y is a linear combination of variables *x*_*i*_(*i* = 1, 2, ⋯⋯*n*), namely:

(2) $$\begin{array}{c} y=b_{0}+b_{1}x_{1}+b_{2}x_{2}+\cdots +b_{n}x_{n} \end{array}$$

In formula (2), *b*_*i*_(*i* = 1, 2, ⋯⋯*n*) denotes the regression coefficient of *i* explanatory variable. For the exchange of (1) and (2), the Logisitic model in terms of occurrence ratio is obtained:

(3) $$\begin{array}{c} Ln\left(\frac{p}{1-p}\right)=b_{0}+b_{1}x_{1}+b_{2}x_{2}+\cdots +b_{n}x_{n}+\varepsilon \end{array}$$

The article "Analysis of Urban Residents' Consumption Behavior and Influencing Factors of Ecological Agricultural Products in the Post-Pandemic Era of COVID-19" was retracted in 2022. Reason: concerns about the peer review.

### 4.2. Variable Description

The dependent variable selected in this article is whether the purchase of multi-ecological agricultural products will increase after the pandemic. According to the hypothesis, seven independent variables were selected as the potential influencing factors of the consumption behavior: the number of family members, family income level, education, gender, age, previous purchase behavior and concerns about agricultural products on the market after the pandemic (see Table 5).

As shown in Table 5, the average number of household members among the surveyed consumers is 2.861, which means most of the surveyed consumers have a family size of between 2 and 4 people; the average family income is 2.455, indicating that the per capita income level is 50,000 to 100,000 yuan per year; the average level of education is 2.204, indicating that the surveyed consumers have a relatively high level of education, with an average of college level or above; the average age is 3.917, indicating that most of the consumers surveyed are between 30 and 50; most people have bought ecological agricultural products; after the pandemic, the average value of safety considerations for agricultural products in the market is 2.435, indicating that after the pandemic, people's attitudes towards agricultural products in the market are between doubt and safe.

### 4.3. Regression Analysis

This paper used the binary Logit regression model to analyze, and the regression results are shown in Table 6.

It can be seen from Table 6 that the regression coefficient of consumers' family members is -0.216, but it does not show significance (z = -1.26, p =0.305>0.05). This means that there is no correlation between family members and consumers' purchase of ecological agricultural products after the pandemic, so Hypothesis 1 has not passed the verification. The size of the family actually reflects the demographic structure of the family, but this does not led to the increase of their purchase of ecological agricultural products after the pandemic. It may be because the size of the family does not change people's ecological awareness, and thus will not affect consumers' future consumption behavior.

The article "Analysis of Urban Residents' Consumption Behavior and Influencing Factors of Ecological Agricultural Products in the Post-Pandemic Era of COVID-19" was retracted in 2022. Reason: concerns about the peer review.

The regression coefficient of the average annual household income level of the consumers is 0.032, which is not significant (z =0.301, p =0.764>0.05), so means that household income has nothing to do with the increase of purchasing ecological agricultural products after the pandemic. The behavior does have an impact, but Hypothesis 2 fails the verification. This may be related to the family's income and expenditure structure, and the expenditure on food for families with higher household income levels is not proportional.

The regression coefficient of consumer education level is -0.210, which does not show significance (z =1.551, p =0.121>0.05). It means that the education level of consumers will not affect people's choice to buy ecological agricultural products, So hypothesis 3 has not been verified. In the survey, the level of education of the consumers are not consistent with their cognition level and consumption ability of ecological agricultural products. The possible explanation is that people with higher education may not play the role of grocery shopping in life, and the activities of cooking and grocery shopping are mainly undertaken by their parents. Therefore, the willingness to consume ecological agricultural products after the pandemic cannot be transformed into the actual purchase behavior of individuals and families.

According to Table 6, gender does not have a significant impact on consumers' ecological agricultural products after the pandemic, and Hypothesis 4 has not not pass the verification. It can be seen from the description that there are more female respondents. Maybe it's due to the fact that women buy agricultural products and cook more frequently than men and they have a better understanding of ecological agricultural products. However, the measurement results show that gender has no effect on the purchase of ecological agricultural products, which may be related to the sampling. As the proportion of male in the sample is relatively low and the ages of the survey are concentrated between 40 and 60, it is impossible to see the significant difference between genders on the purchase of ecological agricultural products.

In the analysis results of age, the regression coefficient is -0.404, showing a significant level of 0.01 (z = -3.486^∗∗^, P =0.000<0.01), which means that age may have a significant negative impact on the purchase behavior of ecological agricultural products. So Hypothesis 5 has been rejected. This shows that older people do not pay more attention to health, nutrition and food safety. Although they are more likely to be responsible for grocery shopping at home, they lack the knowledge of ecological agricultural products. However, young people who have more access to the news about food safety issues may pay more attention to the information of ecological agricultural products. The reasons above have led to the negative influence of age on consumers' purchase of ecological agricultural products.

The article "Analysis of Urban Residents' Consumption Behavior and Influencing Factors of Ecological Agricultural Products in the Post-Pandemic Era of COVID-19" was retracted in 2022. Reason: concerns about the peer review.

The regression coefficient of the option of whether to purchase ecological agricultural products is -0.719, showing a significant level of 0.01 (z =3.885^∗∗^, p =0.003<0.01), which means that people who have bought ecological agricultural products before will not increase the purchase of agricultural products, so hypothesis 6 has been rejected. The possible explanation is that people pay more attention to food safety after the pandemic. People who have not purchased ecological agricultural products before are more willing to purchase ecological agricultural products after the pandemic, while people who have purchased ecological agricultural products before may maintain the previous consumption behavior, showing a negative impact relationship.

The regression coefficient of consumers' attitude towards agricultural products after the pandemic is 0.662, and shows a significance of 0.01 (z =3.885, P =0.000<0.01), which means that the safety of agricultural products has a positive impact on the consumers' purchasing behavior after the pandemic. So Hypothesis 7 has been verified, which shows that consumers who are skeptical of agricultural products in the market after the pandemic have increased their purchases of ecological agricultural products due to food safety considerations.

## 5. Conclusions and Recommendations

### 5.1. Conclusion

This descriptive statistical analysis of data surveyed in this article has shown that: (1) The surveyed consumers had a higher awareness of ecological agricultural products than before; most consumers had bought ecological agricultural products before; consumers were more concerned about the information of ecological agricultural products; most consumers had doubts about the safety of agricultural products after the pandemic. (2) Most of the families were consisted of 3 to 4 members and the people who usually took in charge of purchasing food were mostly middle-aged people between 30 and 59, especially the women. (3) Most people chose to purchase ecological agricultural products in large supermarkets. Moreover, they were willing to get an idea of the supply process of ecological agricultural products, and said that they were willing to spend more to purchase agricultural products to 85.2% when they could understand the traceability of ecological agricultural products, only hoping that the price of ecological agricultural products would not be more than 10% higher, compared with the ordinary agricultural products. (4) The main determinants for consumers to choose ecological agricultural products were safety, nutrition, freshness, price, etc., showing obvious rational consumption characteristics. (5) The consumers did not purchase ecological agricultural products for several reasons: the high price of ecological agricultural products might be the main reason; they were skeptical about the quality of ecological agricultural products; they were in lack of the knowledge of ecological agricultural products.

The article "Analysis of Urban Residents' Consumption Behavior and Influencing Factors of Ecological Agricultural Products in the Post-Pandemic Era of COVID-19" was retracted in 2022. Reason: concerns about the peer review.

The analysis results of the questionnaire under the binary Logit model have shown that: (1) Family members, annual family income, gender, and education level did not affect consumers' consumption behavior of ecological agricultural products after the pandemic. (2) Age and whether consumers have purchased ecological agricultural products before had a significant negative relationship with the consumption behavior of ecological agricultural products. As to age, it's easy to understand that the younger the consumers are, the more they may know about the information concerning food safety during the pandemic, which will affect their consumption concept after the pandemic, being more likely to purchase ecological agricultural products after the pandemic; For those who have bought ecological agricultural products before, they are no strangers to ecological agricultural products, so they will not change the original consumption structure. On the contrary, consumers who have not purchased ecological agricultural products before may be more willing to learn about and purchase ecological agricultural products after the pandemic. (3) There was a significant positive relationship between consumers' attitude and purchase behavior of agricultural products in the market after the pandemic. As consumers who are skeptical of normal agricultural products in the market will increase their purchase of ecological agricultural products after the pandemic.

It should be pointed out that due to the impact of the pandemic, the research coverage of consumption behavior and its influencing factors is limited. So, in the future, we should increase the sample size, expand the regional scope, and take the variables such as consumers' consumption habits and consumption ideas into consideration.

The article "Analysis of Urban Residents' Consumption Behavior and Influencing Factors of Ecological Agricultural Products in the Post-Pandemic Era of COVID-19" was retracted in 2022. Reason: concerns about the peer review.

### 5.2. Recommendations

#### 5.2.1. Vigorously Develop the Integration of Agricultural Socialized Service Industries with Large Supermarkets

Practice has proved that in some places where the development level of the agricultural socialized service industry is relatively high, the impact of the pandemic on agricultural production will be less obvious, and vice versa. The bases of ecological agricultural products are set in the countryside, and the producers of ecological agricultural products are also in the rural areas. The pandemic will inevitably have effect on the production and marketing of ecological agricultural products. So it is necessary to vigorously develop the agricultural socialized service industry, and launch the “order farming” and “contactless farming” programs of ecological products. At the same time, it is essential to connect the agricultural socialized service industry with large supermarkets. The pandemic is both a crisis and an opportunity. Cooperatives are mobilized to participate in social services can improve the service quality, thereby developing an integrated model of production and marketing of social services, which can solve the problems of planting, transportation, and sales of ecological agricultural products during the pandemic, and promote more consumers to purchase ecological agricultural products in large supermarkets.

#### 5.2.2. Improving the Online and Offline Sales Model of Ecological Agricultural Products

Ecological agricultural products are of high prices and uneven quality, which has always been a problem in sales. So, how to make more consumers get an in-depth knowledge about ecological agricultural products is particularly important. In recent years, e-commerce has made a huge contribution to the sales of agricultural products, allowing many consumers to buy low-price and high-quality agricultural products. The sales of ecological agricultural products should follow the same route as agricultural product sales, and adopt a model of simultaneous online and offline sales. The sales of eco-agricultural products should apply the model of “live broadcast from place of origin + online celebrity recommendation”, with particular emphasis on popularizing knowledge of eco-agricultural products, so that consumers can understand and purchase these products. Besides, it is important to expand the scale of production offline and at the same time promote the development of “brother products” through the relevant government sales departments to develop green channels for ecological agricultural products and open up a broader market for ecological agriculture.

The article "Analysis of Urban Residents' Consumption Behavior and Influencing Factors of Ecological Agricultural Products in the Post-Pandemic Era of COVID-19" was retracted in 2022. Reason: concerns about the peer review.

#### 5.2.3. Establish an Ecological Agricultural Product Service Platform

To promote the sales of ecological agricultural products, a multi-level and comprehensive ecological agricultural product service platform, which serves the entire system from top to bottom and from the inside out, should be established. Great efforts should be made to take the lead in realizing a regional ecological agricultural product service platform, which involves farmers, cooperatives, logistics companies, wholesalers. And then it is necessary to realize the connection between regions, the national ecological agricultural product data sharing and unified information, promote the optimization of ecological agricultural products business process, and improve the efficiency of the entire ecological agricultural products. The use of ecological agricultural products service platform can also realize the modern management of the market. Consumers are able to trace the information of the ecological agricultural products they need through the platform, and these information can dispel their doubts about the safety of ecological agricultural products. When more and more consumers are willing to buy ecological agricultural products, producers will be more willing to conduct ecological production behaviors, and the development of ecological agriculture will be enhanced.

#### 5.2.4. Increase Scientific and Technological Research and Application of Ecological Agricultural Products

If the types of ecological agricultural products are limited, and the competition of the ecological agricultural products will be relatively intense. Therefore, we should promote the scientific research on ecological agricultural products and improve the relevant production technologies to enrich their types and give consumers more choices. At the same time, the increasing demand will effectively promote farmers' enthusiasm for planting ecological agricultural products. In order to improve the sustainable progress of ecological agricultural products, the government should make efforts to solve the related technical problems as soon as possible to improve the quality of ecological agricultural products and promote the development of ecological agriculture by customizing and improving the standards of ecological agricultural products.

## Figures and Tables

**Table 1:** Consumer characteristics.

Frequency analysis results				
Title	Options	Frequency	Percentage (%)	Cumulative percentage (%)
Gender	Male	85	19.06	19.06
	Female	361	80.94	100
Age	Under 20	8	1.79	1.79
	20-30 years old	32	7.17	8.97
	31-40years old	82	18.39	27.35
	41-50years old	200	44.84	72.2
	51-60years old	115	25.78	97.98
	Over 60 years old	9	2.02	100
Marital status	Married	404	90.58	90.58
	Unmarried	42	9.42	100
Education level	High school and below	128	28.7	28.7
	Junior college	108	24.22	52.91
	Undergraduate	201	45.07	97.98
	Master degree and above	9	2.02	100
Profession	Farmer	15	3.36	3.36
	Individual merchants	18	4.04	7.4
	Business executives	5	1.12	8.52
	Staff of state-owned enterprises and institutions	292	65.47	73.99
	Private company employees	83	18.61	92.6
	Civil servants	22	4.93	97.53
	Student	11	2.47	100
Total		446	100	100

Note: Data comes from field questionnaire survey.

The article "Analysis of Urban Residents' Consumption Behavior and Influencing Factors of Ecological Agricultural Products in the Post-Pandemic Era of COVID-19" was retracted in 2022. Reason: concerns about the peer review.

**Table 2:** Consumer household characteristics.

Frequency analysis results				
Title	Options	Frequency	Percentage (%)	Cumulative percentage (%)
Family member	1	7	1.57	1.57
	2	73	16.37	17.94
	3 ~ 4	341	76.46	94.39
	5 or more	25	5.61	100
Average family income	Less than 30,000	102	22.87	22.87
	30,000~50,000	129	28.92	51.79
	50,000~100,000	136	30.49	82.29
	100,000 to 200,000	71	15.92	98.21
	200,000~500,000	5	1.12	99.33
	Over 500,000	3	0.67	100

Note: Data comes from field questionnaire survey.

**Table 3:** Consumer Ecological Awareness.

Frequency analysis results				
Title	Options	Frequency	Percentage (%)	Cumulative percentage (%)
Have you heard of ecological agricultural products or green agricultural products?	Yes	419	93.95	93.95
	No	27	6.05	100
How concerned about the information of ecological agricultural products?	Very indifferent	14	3.14	3.14
	Do not care	13	2.91	6.05
	Generally	217	48.65	54.71
	More concerned	137	30.72	85.43
	Very concerned	65	14.57	100
Do you think the food on the market is safe after the pandemic?	Not safe	31	6.95	6.95
	Suspect	198	44.39	51.35
	Safety	209	46.86	98.21
	Very safe	8	1.79	100
Have you bought ecological agricultural products or green agricultural products before?	No	117	26.23	26.23
	Bought	329	73.77	100
Satisfaction after purchasing ecological agricultural products	Null	117	26.23	26.23
	Very dissatisfied	3	0.67	26.91
	Dissatisfied	7	1.57	28.48
	Basically satisfied	218	48.88	77.35
	Quite satisfied	83	18.61	95.96
	Very satisfied	18	4.04	100
Frequency of consumption of ecological agricultural products	Null	117	26.23	26.23
	Buy once in a while	272	60.99	87.22
	Purchase 1 ~ 2 times a week	46	10.31	97.53
	3 purchases a week and above	11	2.47	100
Persons who are mainly responsible for the purchase of agricultural products	Young people under 30	71	15.92	15.92
	30~59 middle-aged people	352	78.92	94.84
	Seniors over 60	23	5.16	100
Total		446	100	100

Note: Null value is a missing data option caused by jump questions.

**Table 4:** Consumer behavior of ecological agricultural products.

Frequency analysis results			
Title	Options	Frequency	Percentage (%)
Where to buy agricultural products before	Hypermarket	291	65.25
	Agricultural market	57	12.78
	Small supermarket	31	6.95
	Others	67	15.02
After the pandemic, will your choice of where to buy agricultural products change?	Yes	118	26.46
	No	328	73.54
After the pandemic, your choice of where to buy agricultural products	Null	328	73.54
	Hypermarket	87	19.51
	Agricultural market	12	2.69
	Small supermarket	9	2.02
	Others	10	2.24
After the pandemic, will you increase your purchase of ecological agricultural products?	Yes	283	63.45
	No	163	36.55
If there is a technology that allows you to understand the supply process of ecological agricultural products, would you like to know this technology?	Willing	342	76.68
	It does not matter	94	21.08
	Unwilling	10	2.24
After you can understand the entire supply process of ecological agricultural products, are you willing to increase your purchase of ecological agricultural products?	Willing	380	85.2
	Unwilling	66	14.8
After the pandemic, how much can you accept that the price of ecological agricultural products is higher than the price of ordinary agricultural products?	10% or less	368	82.51
	11% ~30%	70	15.7
	31% ~50%	8	1.79
Purchase decision factors^∗^	Safety	307	19.08%
	Nutrition	244	15.16%
	Freshness	259	16.10%
	Taste	155	9.63%
	Price	262	16.28%
	Convenient	119	7.40%
	Service	106	6.59%
	Brand	89	5.53%
	Package	68	4.23%

Note: ^∗^ is a multiple choice, so the total number of options exceeds 446; Null is the missing data caused by the data jump.

The article "Analysis of Urban Residents' Consumption Behavior and Influencing Factors of Ecological Agricultural Products in the Post-Pandemic Era of COVID-19" was retracted in 2022. Reason: concerns about the peer review.

**Table 5:** Related variables and mean values.

Variable name	Variable assignment	Mean value	Standard deviation
Family member x_1_	1 person =1; 2 persons =2; 3 ~ 4 persons =3; more than 5 =4	2.861	0.514
Average annual household income x_2_	Less than 30000 =1; 30000~50000 =2; 50000~100000 =3; 100000~200000 =4; 200000~500000 =5; more than 500000 =6	2.455	1.084
Education level x_3_	Below high school =1; college =2; undergraduate =3; master and above =4	2.204	0.882
Gender X_4_	Male =1; female =2	1.809	0.393
Age X_5_	Under 20 years old =1; 21 to 30 years old =2; 31 to 40 years old =3; 41 to 50 years old =4; 51 to 60 years old =5; over 60 years old =6	3.917	0.983
Have you purchased ecological agricultural products X_6_	Bought =1; no =2	1.738	0.44
Consideration on the safety of agricultural products in the market after the pandemic x_7_	Unsafe =1; doubt =2; safe =3; very safe =4	2.435	0.649

**Table 6:** Model analysis of factors affecting consumer choice behavior.

Analysis of binary logit model				
Variable	Regression coefficients	Standard error	z value	p value
Family member	-0.216	0.211	-1.026	0.305
Family income level	0.032	0.106	0.301	0.764
Education level	-0.21	0.135	-1.551	0.121
Gender	0.124	0.271	0.457	0.648
Age	-0.404	0.116	-3.486^∗∗^	0
Have you ever purchased ecological agricultural products	-0.719	0.239	-3.008^∗∗^	0.003
What is your attitude towards market agricultural products after the pandemic?	0.662	0.17	3.885^∗∗^	0
Intercept	1.404	1.1	1.276	0.202
McFadden *R* 方: 0.062				
Cox & Snell *R* 方: 0.078				
Nagelkerke *R* 方: 0.106				

Note: ^∗∗∗^, ^∗∗^, ^∗^ indicate significant at the level of 1%, 5%, and 10%, respectively.

The article "Analysis of Urban Residents' Consumption Behavior and Influencing Factors of Ecological Agricultural Products in the Post-Pandemic Era of COVID-19" was retracted in 2022. Reason: concerns about the peer review.

## Data Availability

The data presented in this study are available on request from Corresponding authors. The data are not publicly available due to privacy.
